# Exploration of the Path of Innovation and Entrepreneurship Education for College Students from the Perspective of Mental Health Education

**DOI:** 10.1155/2022/2659160

**Published:** 2022-04-16

**Authors:** Beibei Wang

**Affiliations:** Zhengzhou University of Industrial Technology, Zhengzhou, Henan 451100, China

## Abstract

Innovation and entrepreneurship education must be based on quality education to train more innovative and high-energy talents, so as to achieve mutual promotion between national development and education reform. The level of college students' psychological quality is the key factor that determines whether they can successfully start a business and succeed. Entrepreneurship requires college students to have the courage and boldness to prevent risks and have the courage and tolerance to face all adverse consequences in the process of entrepreneurship. With the reform of education and teaching in the new era, it has become an inevitable trend to integrate mental health education with entrepreneurship and innovation education in colleges and universities. The development of the country has a greater demand for talents, and colleges and universities are also an indispensable way for talent development and innovation and entrepreneurship education. Combined with the educational practice of contemporary college students, this paper discusses how to promote the integration of mental health education and innovation and entrepreneurship. The educational concept must be innovated in the footsteps of the times so that the two can be organically combined, which is beneficial to the educational cause and can achieve efficient and sustainable development.

## 1. Introduction

In the development of the times, innovation and entrepreneurship education occupies an increasing proportion in contemporary times, so it is necessary to organically integrate innovation and entrepreneurship education with mental health education to help students improve their comprehensive quality as a whole [1]. Innovation and entrepreneurship education must be based on quality education to train more innovative and high-energy talents, so as to realize the mutual promotion between national development and education reform [2]. Although college students' entrepreneurship education and mental health education have their own relatively perfect theories and teaching systems, due to the weakening of psychological counseling in the process of starting a business, more and more students cannot get timely counseling for various psychological problems when starting a business, such as unrealistic, anxiety, fear, and lack of confidence in the face of failure or frustration in starting a business [3]. The level of college students' psychological quality is the key factor that determines whether they can successfully start a business and succeed. Entrepreneurship is a process in which human beings use knowledge and ability to create a career through thinking innovation. Entrepreneurship is a comprehensive test of people's quality, especially the test of people's psychological quality. Entrepreneurial psychological quality refers to the physical and mental organizational elements, structure, and quality level formed and developed under the influence of environment and education and fully and stably displayed and played a role in entrepreneurial social practice; it is a characteristic of personality consciousness that regulates people's psychology and behavior. It can not only refer to the entrepreneurial psychological quality potential to be developed in people's quality but also refer to people's entrepreneurial psychological quality that has been internalized. It can refer to both individual entrepreneurial psychological quality and group entrepreneurial psychological quality. Good entrepreneurial psychological quality is like the cornerstone of entrepreneurial building, which can lay the foundation of career and support entrepreneurial life. Entrepreneurship requires college students to have the courage and boldness to prevent risks, and have the courage and tolerance to face all adverse consequences in the process of entrepreneurship [4]. Promoting the integration of mental health education in colleges and universities with the concept of “double innovation” education is one of the main tasks of mental health theory courses in colleges and universities at present [5]. Innovation and entrepreneurship ability is the ability of college students to adapt to the development requirements of the times, and it is a new survival skill in the new period. To enhance their innovation and entrepreneurship ability, we must create a good atmosphere of innovation and entrepreneurship and build a perfect innovation and entrepreneurship cultivation system [6].

With the reform of education and teaching in the new era, it has become an inevitable trend to integrate mental health education with entrepreneurship and innovation education in colleges and universities. The development of the country has a greater demand for talents, and universities are also an indispensable way for the development of talents, innovation, and entrepreneurship education [7]. As the cradle of education, colleges and universities are the base for cultivating innovative talents. Promoting the popularization of innovation and entrepreneurship education for college students can not only provide powerful assistance for the reform of market structure but also meet the basic requirements of socialist modernization [8]. Colleges and universities are important places to carry out mental health education and cultivate innovative and entrepreneurial talents. Mental health education is a practical activity to carry out Marxist education, ideological education, and moral education. Innovation and entrepreneurship education is education from imparting knowledge to creating knowledge and from reserving knowledge to activating knowledge [9]. Innovation and entrepreneurship activities are more a test of students' psychological quality. When students have strong entrepreneurial psychological quality, it means that they have the cornerstone of the entrepreneurial building [10]. Innovative entrepreneurs should continue to learn, never relax the cultivation of their own abilities, and, at the same time, have solid professional knowledge and skills [11]. Both have the same value orientation and academic basis, and the innovation and entrepreneurship education and mental health education have the same goal, the same content, and compatible methods [12].

For the teaching work of any subject, if we want to continuously enhance its influence, we should not only pay attention to the integration of advanced educational concepts but also meet the educational development needs of the times [13]. Mental health education is an important way for college students to cultivate innovative consciousness and spiritual civilization. Incorporating innovation and entrepreneurship education can not only improve the innovation enthusiasm of college students but also have a good practical significance for promoting scientific and technological innovation and economic construction [14]. If innovation and entrepreneurship education wants to develop well, it cannot be separated from mental health education in colleges and universities. Only by establishing correct ideological values for college talents can it provide guarantee for the sustainable development of their abilities in all aspects [15]. At present, China is in a critical period of building a well-off society in an all-round way and accelerating modernization, and high-quality talents are the main reserve force for promoting social development [16]. Mental health education and innovation and entrepreneurship education complement each other and penetrate each other. It is very necessary to study the organic integration of mental health education and the cultivation of innovative and entrepreneurial talents [17]. Combining with the educational reality of contemporary college students, this paper discusses how to promote the integration of mental health education and innovation and entrepreneurship. The educational concept must be innovated in the footsteps of the times so that the two can be organically combined, which is beneficial to the educational cause and can achieve efficient and sustainable development.

## 2. Promoting Effect of Mental Health Education on Innovation and Entrepreneurship Education in Colleges and Universities

### 2.1. Stimulating the Enthusiasm of Innovation and Entrepreneurship

As the key content of psychological education, mental health knowledge is very important to improve students' psychological quality. To a certain extent, psychological quality education can influence students' establishment of outlook on life, maturity of personal thoughts, and adaptability to social environment. The new era is one that emphasizes mass entrepreneurship and innovation. The development of higher education should keep pace with the times and develop the same frequency resonance at the same time. There is an inevitable connection between mental health education and innovation and entrepreneurship education in colleges and universities. With the development of education, it is imperative to integrate them [18]. Therefore, in the integration of the two, a certain foundation is needed to provide the possibility for the integration of the two. At present, many people begin to pay attention to quality education, but quality education is still based on examination-oriented education. In the examination-oriented education for many years, students' thinking has been solidified, and most of them have the same thinking form, lacking innovation and diversity. In the field of psychological education, mental health knowledge is a very important content. Implementing mental health education and enriching students' mental health knowledge plays a vital role in improving college students' psychological quality [19]. The training mode of collaborative education can better realize the integration of the two, guide students in the teaching process, deepen their ideological understanding, improve their cognitive level, and guide students to establish a correct view of employment and entrepreneurship. At the same time, it can also help students establish a sense of responsibility of active innovation and courage, which is helpful to improve the quality of higher education personnel training.

Innovation-driven economies score higher than investment-driven economies in entrepreneurship policy. This is mainly due to the higher level of economic development driven by innovation, the more perfect policy system, and the higher efficiency of the allocation of entrepreneurial resources.  Figure 1 is a conceptual model of the mechanism of the influence of entrepreneurship policy on entrepreneurs' entrepreneurial behavior.

Employment competitiveness is the ability of individuals to obtain and keep jobs, make progress in their jobs, and cope with changes in their work and life. The concept of employment is not static, but developing constantly. With the change of environment, economic status, and outlook on life and private world, this concept will change accordingly. This paper makes statistics on the survey results of the degree of management education objectives when some college courses achieve entrepreneurial awareness. There are many factors that make it difficult for college students to find jobs.  Table 1, for example, is the survey and statistics on the degree of management education goals when curriculum teaching realizes entrepreneurship awareness.

College students' mental health education is to set a correct direction for the development of students' thoughts, behaviors, and qualities, and to educate students' political literacy, ideological qualities, life values, mental health, and related legal awareness. A simple and effective method to analyze the differences between mental health education and vocational skills training is hypothesis testing of two independent sample methods. In the student evaluation, the evaluation data of teachers are shown in Table 2.

Faced with entrepreneurship, students often have great pressure and fear, which directly affect the courage and motivation of entrepreneurs. College students need to complete the transformation from students to social people after graduation, and the change of environment has brought about some changes in their hearts. The emergence of these negative psychological emotions will directly affect their normal life and will also have a negative impact on their innovation and entrepreneurship development [20]. Therefore, college students must eliminate this unhealthy psychology in time and actively learn some knowledge about mental health before entering the workplace. In terms of curriculum, mental health education and innovation and entrepreneurship education are independent, and there is no intersection. To a certain extent, psychological quality education will more or less affect college students' establishment of outlook on life, which is related to the maturity of their personal thoughts and their ability to adapt to the environment in society. Therefore, in the process of college education and teaching, we should pay attention to the education and teaching of college students' mental health, effectively dig out the connotation and essence of mental health education, better enhance the comprehensive ability of college students, and promote the improvement of students' self-education ability, thus providing the premise and foundation for college students to innovate and start businesses after graduation.

### 2.2. Improving Psychological Quality

The mutual promotion and integration between mental health education and innovation and entrepreneurship education are of great value to the cultivation of talents in colleges and universities. The innovation of educational methods has been achieved both in theory and in practice, which really meets the needs of students' career development. Mental health education is the basic education of all education, which provides a better platform and space for students' all-round development. On the surface, innovation and entrepreneurship education is to cultivate students' innovative consciousness to enhance their entrepreneurial ability, to establish a correct concept of entrepreneurship and employment for their personal development, and to make students better adapt to social life [21]. The scientific integration of the two educational concepts requires both theoretical basis as a guide and practical basis as a reference. From the perspective of the integration and development of mental health education and “double innovation” education in colleges and universities, the two bases are quite sufficient.

Systematic psychological training plays a vital role in improving college students' psychological skills. We should study the present situation of college students' psychological training. In addition to the research of training methods and means, we should also investigate the formulation of their psychological training plans. For example, Table 3 shows the investigation of psychological training plan.

Health is not only the absence of disease and weakness but also the physical, psychological, and social perfection. When constructing the base classification, it is necessary to comprehensively consider the storage and time overhead allowed in practical applications to select the appropriate integration scale as shown in Figure 2.

Because the establishment and maintenance of social relations need certain emotional and spiritual support, if entrepreneurs have effective social relations, it is also emotional guarantee for entrepreneurial activities and then enhances their entrepreneurial performance. For example, Table 4 shows the empirical analysis results of entrepreneurship policy and entrepreneurship strategy.

In order to eliminate the influence of different dimensions of original data, data preprocessing is based on data mining. Standardized formula is as follows:

(1) $$\begin{array}{c} {\text{CI}}_{i}=\frac{\sum_{j}\left(C_{ij}/C/N\right)\ln\left(C_{ij}/C/N\right)}{N\;\ln\left(N\right)}. \end{array}$$

Need to meet the following:

(2) $$\begin{array}{c} P_{i}=\frac{f_{i}}{\sum_{i=1}^{N}f_{i}}. \end{array}$$

Define the distance formula as follows:

(3) $$\begin{array}{c} Y_{j}\left(t\right)=\phi \left(\sum_{i=1}^{n}w_{ji}x_{i}-\theta_{j}\right). \end{array}$$

Take the variance contribution rate of each factor as the weight and take the first *n* factors to reflect the original evaluation index

(4) $$\begin{array}{c} o_{j}\left(t\right)=f\left(\left[\sum_{i=1}^{n}w_{ij}x_{i}\left(t-\tau_{ij}\right)\right]-T_{ij}\right). \end{array}$$

Entrepreneurship funding system can help individuals develop entrepreneurial opportunities, entrepreneurship education system can improve entrepreneurs' ability to identify opportunities, and the optimization of entrepreneurial environment will provide entrepreneurs with more entrepreneurial opportunities. For example, Table 5 shows the empirical analysis results of entrepreneurial policy and entrepreneurial attitude, and Table 6 shows the empirical analysis results of entrepreneurial policy and entrepreneurial mode.

In mental health education, teachers should know the students' psychological changes in time and arouse their enthusiasm for innovation and entrepreneurship in many ways, which can not only effectively enhance their self-education ability but also reduce innovation and entrepreneurship as their future study and development direction [22]. We should pay attention to the mental health education of college students, deeply explore the essence and connotation of education, improve students' comprehensive ability and self-education ability, and lay the foundation for cultivating college students' innovation and entrepreneurship. At the same time, teachers should understand students' psychological dynamics, stimulate their enthusiasm and enthusiasm for innovation and entrepreneurship, and let them take innovation and entrepreneurship as their motivation and development direction while improving their self-education ability. Only by cultivating talents with excellent comprehensive quality can we perfect and even optimize the structure of human resources in society and then promote the development of social economy.

## 3. The Path of Entrepreneurship Education for College Students from the Perspective of Mental Health Education

### 3.1. Optimizing the Curriculum

In the innovation and entrepreneurship education of colleges and universities, the mental health education of college students is very important. Only when college students have a healthy psychological quality can they carry out innovation and entrepreneurship better. There is a close relationship between mental health education and entrepreneurship education in colleges and universities. Therefore, under the background of educational reform in the present era, specific measures need to be implemented to promote the effective combination of innovation and entrepreneurship education in mental health education in colleges and universities. There is a disconnect between mental health and innovation and entrepreneurship education courses in colleges and universities, so introducing mental health education into innovation and entrepreneurship education courses is beneficial to students' psychological quality [23]. If we want to promote the organic integration between mental health and innovative education in colleges and universities, we must first improve the cohesion mechanism of their classroom contents, so as to achieve mutual reference between their contents and ideas. Most innovation and entrepreneurship education did not pay attention to the theory of mental health in political education and did not apply the theory and innovative knowledge to practice, ignoring the cultivation of moral quality and ideological literacy, which made it difficult to integrate mental health with innovation and entrepreneurship.

For students with psychological problems, it is necessary to set up psychological health personal files, find out the causes of psychological problems in time, and give correct guidance and treatment to the problems so that students can treat mental health problems correctly, thus helping them to establish mental health awareness and enhance social adaptability. Only by understanding the employment concept of college students can the education and teaching management, mental health education, and employment guidance in colleges and universities be more targeted, so as to better carry out the education of employment outlook.  Figure 3 shows the dynamic evolution of the evaluation system of college students' entrepreneurial awareness.

Mental health education in colleges and universities has been explored and practiced for decades, but the foundation of innovation and entrepreneurship education is weak at the beginning, and the teaching methods and modes need to be improved. For innovation and entrepreneurship, the foundation of practice and exploration is also weak [24]. Mental health in colleges and universities and innovation and entrepreneurship education of college students are quality education, which have solved the value orientation and innovation problems of contemporary college students well. For practical activities, they are related to each other. From the aspect of maximizing value, only by doing a good job of exploration can we improve the effectiveness of education. In the process of classroom teaching, teachers should take students as the main body, such as performing psychological sitcoms with the theme of innovation and entrepreneurship so that students can experience the inner activities and emotional experiences of entrepreneurs so that they can better understand entrepreneurship and actively experience entrepreneurship.

### 3.2. Improving Psychological Tools

Strengthening psychological counseling for innovative and entrepreneurial students can help them to carry out entrepreneurial activities more effectively. In the process of innovation and entrepreneurship, we can combine the characteristics of college students and different stages of the university and carry out corresponding psychological counseling for entrepreneurship, so as to inspire students and make them learn to adjust themselves. To implement the integration requirements of mental health and innovation and entrepreneurship education, we must start with practice and set up an effective practice platform for students. First, stimulate the carrier function of community. Teacher training is a key factor for the organic integration of mental health education and innovation and entrepreneurship education in colleges and universities. The organic combination of the two lies in the guidance of relevant educators to a great extent. The characteristics and essence of innovation and entrepreneurship determine the community entrepreneurship activities in colleges and universities. Taking the community as the basis, we can improve the creativity and enthusiasm of members through mutual help, encouragement, and respect. Of course, this is the value pursuit of innovation and entrepreneurship education and mental health education [25]. There is only a certain degree in the two kinds of education for college students. Therefore, educators engaged in the related education should strengthen the communication and cooperation in teaching content and objectives in practical work, so as to better promote the organic integration between the two. The integration of innovation and entrepreneurship with mental health education must be put into practice. By improving the flexibility of acceptance, we should do a good job in publicizing innovation and entrepreneurship, and then put it into practice. For those college students who have strong entrepreneurial motivation and entrepreneurial strength, we should carry out targeted entrepreneurship psychological education, improve students' entrepreneurial psychological quality through entrepreneurship psychological education, and better deal with various problems in the process of entrepreneurship.

### 3.3. Strengthening the Construction of Teachers

Whether it is mental health or innovation and entrepreneurship education, it is necessary to do a good job as an education leader and make use of teachers who are brave in innovation and excellent in quality to integrate the two. For the occurrence of mental health problems of college students, mental health education teachers should make early detection and prevention, so as to effectively control the occurrence and development of mental health problems. Therefore, it is necessary to investigate the mental health of college students as soon as possible, so as to know the changes of students' mental state in time, and make a health education plan in a planned and targeted way according to students' personality characteristics, and put the health education plan into practice. In the innovation and entrepreneurship education, teachers must have the spirit of self-motivation and innovation, so as to constantly strengthen their beliefs and improve students' innovative spirit. In the process of curriculum implementation, the content of books is only one of the educational resources, and more teaching content needs teachers to dig deeply by relying on the Internet and modern educational technology, and set entrepreneurial topics for students so that students can imitate successful cases of entrepreneurship. Innovation and entrepreneurship have rich practice and profound theoretical spirit, as well as the ability of management and moral cultivation, which are infiltrated into the teaching staff, and entrepreneurial innovation is set up on the background of mental health education. As far as higher education is concerned, teachers play an important role in the transmission of knowledge, the shaping of consciousness, and the cultivation and guidance of quality and ability. Teachers should give priority to guidance in teaching philosophy and play the role of the main channel in classroom teaching.

## 4. Conclusion

To carry out innovation and entrepreneurship education in colleges and universities, it is necessary to cultivate college students' innovative ability and awareness and improve their psychological quality. In the work of college students' innovation and entrepreneurship education, it is necessary to cultivate college students' innovative consciousness and ability in a planned way, and improve their psychological quality from various aspects. Only by maintaining good psychological quality can college students resist the influence of various external factors in the complicated social competition environment. In the new era of education in China, the integration of mental health education and innovation and entrepreneurship education has become the general trend. Therefore, although colleges and universities have made a breakthrough in the organic integration of mental health education and innovation and entrepreneurship education, they still cannot relax, and we need to pay close attention to the trend of education reform. In the process of innovation and entrepreneurship, only by maintaining good psychological quality can we resist the interference of various adverse factors in the complex society, face all kinds of setbacks and difficulties, establish self-confidence in the success of entrepreneurship, and constantly enhance its ability of innovation and entrepreneurship. To implement the development strategy, colleges and universities must take the responsibility of education and integrate the two together based on the realistic background, so as to achieve the goal of economic, convenient, and efficient personnel training.

## Figures and Tables

**Figure 1:** Conceptual model of the influence mechanism of entrepreneurial policy on entrepreneurs' entrepreneurial behavior.

**Figure 2:** Influence of different integration scales on the accuracy of college students' psychological behavior operation.

**Figure 3:** Dynamic evolution of the entrepreneurial awareness evaluation system.

**Table 1:** Investigation on the degree of teaching to achieve the goal of entrepreneurship awareness and management education.

Degree of realization	Fully realized	Partially realized	Not implemented
Selected number of people	28	56	52
Proportion (%)	20.1	41.2	38.2

**Table 2:** Student evaluation data of two independent sample means.

Sample size	Average score	Sample standard deviation
42	79	4.2
42	72	3.7
43	81	4.8

**Table 3:** Investigation of psychological training plan.

	Number of people	Proportion (%)
Make a systematic psychological training plan	22	11
Arrange according to experience	178	89

**Table 4:** Empirical analysis results of entrepreneurial policy and entrepreneurial strategy.

Variable	Scale expansion	Internationalization expansion
Entrepreneurial support	0.082	0.083
Entrepreneurship education	0.074	0.066
Entrepreneurial environment	0.052	0.269
Type of economy	0.538	0.237

**Table 5:** Empirical analysis results of entrepreneurial policies and entrepreneurial attitudes.

Variable	Perceptual skills	Perceived opportunity	Entrepreneurial willingness	Fear of failure
Entrepreneurial support	0.079	0.155	0.071	0.271
Entrepreneurship education	0.068	0.257	0.065	0.395
Entrepreneurial environment	0.024	0.095	0.059	0.026
Type of economy	0.026	0.087	0.095	0.036

**Table 6:** Empirical analysis results of entrepreneurial policies and entrepreneurial models.

Variable	Survival entrepreneurship	Opportunity-based entrepreneurship
Entrepreneurial support	0.351	0.288
Entrepreneurship education	0.257	0.165
Entrepreneurial environment	0.088	0.178
Type of economy	1.471	2.547

## Data Availability

The data used to support the findings of this study are included within the article.

## References

[1] Li X. (2017). Innovative mental health education to promote the development of innovation and entrepreneurship education in colleges and universities. *Quality Education in West China*.

[2] Zhang Y. (2019). Research on the integration of ideological and political education and innovation and entrepreneurship education in colleges and universities. *Science and Technology of Energetic Materials*.

[3] Peng F. (2018). Research on the path of integrating ideological and political education into innovation and entrepreneurship education in colleges and universities. *Journal of Social Sciences of Jiamusi University*.

[4] Lei Y. (2018). The path of integrating ideological and political education into innovation and entrepreneurship education in colleges and universities. *Journal of Donghua University*.

[5] Zhao X. (2018). Ideological and political education and innovation and entrepreneurship education. *Think Tank Times*.

[6] Liu Y., Cai H. (2016). Research on the integration of entrepreneurship education and ideological and political education in colleges and universities. *Journal of Hebei University of Technology: Social Science Edition*.

[7] Zhang C. (2019). Discussion on network mental health education for college students based on “Internet+”. *Research and Practice on Innovation and Entrepreneurship Theory*.

[8] Suseno Y., Abbott L. (2021). Women entrepreneurs’ digital social innovation: Linking gender, entrepreneurship, social innovation and information systems. *Information Systems Journal*.

[9] Qian Y. (2020). Research on the psychology of innovation and entrepreneurship of students majoring in film and television media in higher vocational colleges. *Journal of Hubei Correspondence University*.

[10] Li D. (2020). Exploration and attempt to carry out mental health and entrepreneurship education for freshmen in colleges. *Farm Staff*.

[11] Rong Y. (2019). Strategies for constructing a psychological support system for college students’ innovation and entrepreneurship under the new situation. *Journal of Anshan Normal University*.

[12] Qin J. (2017). Analysis of the causes of postgraduate mental health problems under the background of innovation and entrepreneurship. *Science & Technology Monthly*.

[13] Xiao Q. (2019). Construction of teacher competency model for mental health education in vocational colleges. *Research and Practice on Innovation and Entrepreneurship Theory*.

[14] Wang D. (2019). Research on the mutual promotion of ideological and political education and innovation and entrepreneurship education in colleges and universities. *Journal of Weifang Engineering Vocational College*.

[15] Xia H. (2020). Research on the coordinated development path of ideological and political education and innovation and entrepreneurship education in colleges and universities under the new situation. *Journal of Hubei Correspondence University*.

[16] Ao Y., Zhang Z. (2019). The integration of ideological and political education and innovation and entrepreneurship education in colleges and universities. *Journal of the Party School of Shanxi Provincial Committee of the Communist Party of China*.

[17] Zhang W. (2019). Research on ideological and political education helping the development of innovation and entrepreneurship education. *Think Tank Times*.

[18] Yang Z. (2018). Research on the collaborative education model of ideological and political education and innovation and entrepreneurship education. *Journal of Jilin Teachers College of Engineering and Technology*.

[19] Cui L. (2018). Research on the promotion of innovation and entrepreneurship education by ideological and political education in colleges and universities. *New West*.

[20] Jin C. (2020). Analysis on the mental health education strategy of undergraduates’ entrepreneurship from the perspective of positive psychology. *Innovation and Entrepreneurship Education*.

[21] Sun Y. (2017). Research on university innovation and entrepreneurship education from the perspective of psychological capital. *Quality Education in West China*.

[22] Aly M., Audretsch D. B., Grimm H. (2021). Emotional skills for entrepreneurial success: the promise of entrepreneurship education and policy. *The Journal of Technology Transfer*.

[23] Gouvea R., Kapelianis D., Montoya M. J. R., Vora G. (2021). The creative economy, innovation and entrepreneurship: an empirical examination. *Creative Industries Journal*.

[24] Wu S., Jiao D. (2019). Research on the application of mental health education in the employment and entrepreneurship education of college students under the background of we-media. *Theoretical Research and Practice of Innovation and Entrepreneurship*.

[25] Tian S. (2016). Research on health education based on college students’ fear of starting a business. *Liaoning Economics*.

